# Groundwater Suitability Evaluation Using Entropy Weightage Quality Index (EWQI) Model and Human Health Cancer Risk Assessment of Heavy Metal in Eastern India

**DOI:** 10.1155/2022/2476126

**Published:** 2022-07-12

**Authors:** Shivam Saw, Prasoon Kumar Singh, Jaydev Kumar Mahato, Rohit Patel, Deepak Naresh Dhopte, Evans Asenso

**Affiliations:** ^1^Department of Environmental Science and Engineering, IIT (ISM), Dhanbad, Jharkhand, India; ^2^Department of Agricultural Engineering, University of Ghana, Ghana

## Abstract

This study evaluated the groundwater using the Entropy Weightage Quality Index model (EWQI). Eighteen samples were taken from the different wellbores during premonsoon seasons in 2021. The present study is aimed at developing a comprehensive approach for groundwater quality assessment and associated health risk along with the cancer risk due to the presence of heavy metals. The water quality of Ranchi city was found to be better except in the western zone. Principal component analysis (PCA) revealed that arsenic (As) was the most influencing element that deteriorated the potability of water which supports our study. The study looked at cancer and noncancer health hazards connected with heavy metal music. The value of hazardous quotient (HQ) was observed to be relatively higher in As (HQ > 1) and Ni, followed by Mn > Fe > Zn > Cu. Also, the children were at higher risk than adults. The cancer risk associated with arsenic was investigated and found that the northern part and southeast-west (lapung block) of the study are at higher risk. Prolonged ingestion of As causes diseases like arsenicosis that leads to enhanced chances of cancer risk. This research provides an immense research database to assess the potability of drinking water in a similar city like Ranchi.

## 1. Introduction

Globally, it has been considered that groundwater is an essential natural reserve for the existence of life, and approx. two billion people worldwide rely on it [1]. India is heavily reliant (25%) on groundwater resources, followed by the United States (11%) and China (11%). Among all the consumption activities, nearly 85% of the supply is consumed for drinking purposes and 60% for the agricultural activities [2]. During 2013-14 to 2019-20, the Indian government has launched a potable water supply and cleanliness program for low-income states, such as Jharkhand in association with the world bank. The wells and bore wells are vital resources for drinking water in a rural area of this state. Contamination and degradation of groundwater can occur naturally by the interlinkage of hazardous materials found in topsoil and rocks beneath the earth's surface, and contamination can occur artificially by the activity of poor drainage systems, agriculture, discharge of untreated sewage, and industrial water [3, 4]. This contamination mechanism in groundwater varies widely on the basis of landuse pattern, lithological characteristics water-rock-soil interrelation, physicochemical excellence, microbial and mineral existence, and other factors [5]. Land use and lithological characteristics interrupt groundwater resources through changes in recharge and by altering demands for water. Inappropriate land use, primarily poor land management, causes chronic groundwater quality problems. Human health is jeopardized by the presence of harmful elements in groundwater sources. These elements are nonbiodegradable, immobile, poisonous, and bioaccumulative, with a thousand-year residence duration. Recently, there has been a lot of focus on evaluating the chemical parameters of potable water and the related health problem linked with nitrate (NO3^−^) and fluoride (F^−^), which are considered to be the most prevalent chemical elements and also found to be most toxic [6–8]. Li et al. [9] investigated the groundwater quality and its risks posed by pollutants such as nitrate and fluoride ions in an arid climate zone near northwest China, and the study reported that responsible pollutants emerge from industrial, agricultural, and geogenic sources. They also discovered that adults are not as vulnerable to health risks as children and girls. The hazard in respect of both carcinogenic and noncarcinogenic impacts can be assessed using human health risk assessment [10]. Kaur et al. [11] investigated the impact of human interventions on drinking water in Panipat, India, and the subsequent impact on the health of the exposed people, finding that kids are at a higher danger as compared to men and women cases of noncarcinogenic risk. The application of entropy approaches to the weighting of each assessment index is a very relative technique that successfully removes human prejudices. In India, various studies evaluate the quality of drinking water for irrigation and consumption in Andhra Pradesh (Subba Rao et al. [4]), Chandigarh (Rahman et al. [12]), and various parts of the country. Water polluted with As (arsenic) has caused major chronic human ailments such as dermatological disorders, arsenicosis, keratosis, and cancer all over the world [12]. In 2005, the National Metallurgical Laboratory in collaboration with United Nations International Children's Emergency Fund (UNICEF) confirmed the existence of arsenic in Sahibganj [13].

Ranchi, the state capital of Jharkhand, is emerging as a major educational and industrial center. Because of the reason of involuntary development, movement of people from rural to urban areas, insufficient drainage systems, and inefficient sewage disposal services in various major and small-size companies, and periurban accumulation are deteriorating in most Indian towns [14]. As a result, strong water management is essential to meeting basic water needs; otherwise, substantial environmental and health costs will be incurred. Efficient water management requires accurate assessment and investigation of drinking water quality. Several indices of water quality can aid in handling enormous volumes of water quality data because they are an excellent method for condensing huge quantities of data into a single numeric number allowing for a simple and easy explanation of the observed data [15]. Conducted a study for evaluation of only the quality of groundwater resources in Zanjan Plain using EWQI. Adimalla [16] conducted a study in the rural area of Telangana state, India, to assess the groundwater quality using EWQI and pollution index. Kumar and Augustine [17] carried out the assessment of groundwater quality of Odai Sub-Basin, South India. Such previous studies were limited to the assessment of groundwater quality incorporating EWQI approach, but the present study comprises of comprehensive approach for groundwater quality assessment and associated health risk along with the cancer risk due to presence of heavy metals in eastern India.

The goal of this work was to assess (i) spatial distribution analysis to determine the overall acceptability of groundwater quality using an entropy-weighted water quality index (EWWQI), (ii) hazard index (HI), to carry out the risk associated with drinking water for the residents who are using extremely contaminated groundwater for drinking purposes, (iii) the carcinogenic risk assessment of arsenic, and (iv) principal component analysis (PCA) and hierarchical cluster analysis of the study area. This research contributes to the identification of the intensity of distinct zone of vulnerability at a particular location to adopt effective methods to enhance groundwater quality.

## 2. Materials and Methods

### 2.1. Location Map of Study Area

In present study, all the samples were collected from Ranchi, Jharkhand, during April-May month of 2021. It is situated at 23.37°N latitude and 85.35°E longitude, and its height is about 2300 feet above sea level. According to the census of Ranchi Municipal Corporation (RMC) 2011, it has a total population of around 1,073,440. The average annual rainfall of Ranchi is 1394 mm. The water sample was collected from the 18 defined groundwater wells of Ranchi city. The location sites were selected at random based on the availability of wells (Figure 1). ArcGIS, version 10.3, was used to create the sampling sites and spatial distribution maps. The methodology involved in the present study is shown in the form of flow diagram in Figure 2.

### 2.2. Computational Methods

The physicochemical properties of groundwater samples were calculated in their entirety as per the standards protocol of APHA [18]. The value of pH and electrical conductivity (EC) was evaluated on the site using water quality multimeter (Model No. Hach HQ430d). Cations (Na^+^, K^+^, Ca^2+^) were analyzed by using flame photometry (Model 1385), while the anions i.e., sulfate (SO_4_^2-^), chloride (Cl^−^), and fluoride (F^−^) are done by using the turbidimetric method, argentometric method, and SPADNS methods, respectively. The heavy metal concentration was analyzed by atomic absorption spectrophotometry (AAS) (REF-3000AA, Refinement). In this case, the widespread use of AAS across the globe is ascribed to its acceptance, recognizability, usability, and affordability when compared to other fundamental approaches like inductively coupled plasma. Additionally, AAS is a sensitive technique that may identify elements at quantities as low as ng/mL, particularly when using the graphite furnace mode for atomization. Due to the use of a selective irradiation source, AAS also benefits from good selectivity. Excel 2019 and Origin software version 20 were used to conduct the statistical analysis.

### 2.3. Entropy-Weighted Water Quality Index (EWWQI)

The EWWQI is a scientific tool for determining quality for drinking purposes and other domestic uses [19, 20]. The calculation procedures of EWWQI consist of 5 different steps [21, 22] which are as follows.

The matrix (*A*) is an eigenvalue matrix connected with water quality information for “*m*” no. of various samples and “*n*” no. of physicochemical parameters during the first step (Eq. (1)).

(1) $$\begin{array}{c} \text{A}=\left|\begin{array}{ccc} a_{11} & a_{12} & \cdots a_{1n}\\ a_{21} & a_{22} & \cdots a_{2n}\\ a_{m1} & a_{m2} & \cdots a_{mn} \end{array}\right|. \end{array}$$

The above matrix (*A*) was modified into a new-grade matrix (*B*) in the second stage, using Equations (2) and (3).

(2) $$\begin{array}{c} b_{ij}=\frac{a_{ij}-\left(a_{ij}\right)\min}{{\left(a_{ij}\right)}_{\max}-{\left(a_{ij}\right)}_{\min}}, \end{array}$$

(3) $$\begin{array}{c} \text{B}=\left|\begin{array}{ccc} b_{11} & b_{12} & ..b_{1n}\\ b_{21} & b_{22} & ..b_{2n}\\ b_{m1} & b_{m2} & ..b_{mn} \end{array}\right|. \end{array}$$

The information entropy (ej) was calculated in the third stage, using Equations (4) and (5).

(4) $$\begin{array}{c} e_{j}=-\frac{1}{Inm}\overset{m}{\underset{i=1}{\sum }}\;P_{ij}\text{In}P_{ij}, \end{array}$$

(5) $$\begin{array}{c} P_{ij}=\frac{\left(1+b_{ij}\right)}{\sum_{i=1}^{m}\;\left(1+b_{ij}\right)}. \end{array}$$

Using Equations (6) and (7), the weight of entropy (wj) and the rating scale (qj) were evaluated in the fourth step.

(6) $$\begin{array}{c} w_{j}=\frac{\left(1-e_{j}\right)}{\sum_{i=1}^{m}\;\left(1-e_{j}\right)}, \end{array}$$

(7) $$\begin{array}{c} q_{j}=\frac{C_{j}}{S_{j}}\times 100. \end{array}$$

According to WHO [23] and BIS [24], *C*_*j*_ is the physicochemical parameter (*j*) content (mg/L), and *S*_*j*_ is the standard desired limit of the physicochemical parameter (*j*) given in mg/L. Finally, EWWQI was calculated with the help of equation (8).

(8) $$\begin{array}{c} \text{EWWQI}=\overset{m}{\underset{j=1}{\sum }}\;w_{j}q_{j}. \end{array}$$

With the help of EWQI modeling approach different categories are assigned corresponding to EWQI range, excellent quality has been assigned to the EWQI if it is below 25, the good quality between 25 and 50, medium quality between 50 and 100, poor quality between 100 and 150, and unfit for drinking if it is above 150. Additionally, Table 1 presents the EWQI rankings and classification for groundwater quality [25].

### 2.4. Health Risk Assessments of Heavy Metals

The noncarcinogenic human health risk due to the oral exposure associated with the heavy metals present in groundwater was evaluated by the computation of total hazard index (HI) given by methods (Eq. (9)). The noncancer risks were characterization as hazard quotient (HQ) (Eq. (10)). It is the ratio of individual element exposure levels to the reference dose (RfD) of the corresponding element. The RfD values of various heavy metals are based on the hazard index (HI) value, which is the ratio of multiple substance/unit-exposure pathways and can be expressed as the sum of all HQ values (Eq. (11)).

(9) $$\begin{array}{c} \text{ADD}=\left(\text{Cw}\times \text{Ir}\times F_{R}\times E_{D}\right)/\left(W_{b}\times Tm\right), \end{array}$$

(10) $$\begin{array}{c} \text{HQ}=\text{exposure level}\frac{\left(\text{ADD}\right)}{\text{RfD}}, \end{array}$$

(11) $$\begin{array}{c} HI=\sum \text{H}\text{Q}. \end{array}$$

Here, ADD is the mean daily dose of heavy metals (mg/kg/day), *C*_*W*_ is the concentration of heavy metals (mg/l) in the water samples, Ir is the rate of ingestion (3 l/day for adults), *F*_*R*_ is the frequency of exposure (days/year), *E*_*D*_ is the total duration of exposure (years), *W*_*b*_ is the average weight of (60.5 kg in adults) [10], and Tm is the meantime (days).

The product of ADD (mg/kg/day) and SF (mg/kg/day/)-1 was used to determine the carcinogenic hazard. The characterization scale was derived using Table 2 as a guide [26].

## 3. Result and Discussion

### 3.1. Physicochemical and Hydrogeochemical Characterization of Groundwater

Table 3 shows the summary data regarding the physicochemical quality of groundwater in Ranchi. The pH value was observed mostly basic in nature that varied from (7 to 8.1). The measured value of electrical conductivity (EC) in the study area varies from 236 to 1369 *μ*S/cm. The chemistry of cations in the study has the dominancy of calcium (Ca^2+^) > magnesium (Mg^2+^) > sodium (Na^+^) and > (potassium) K^+^. In contrast, the observed seasonal value of anions was the highest in bicarbonate (HCO_3_-) and lowest in fluoride (F^−^). The geochemical processes and interactions of numerous minerals and organic materials are the fundamental causes of variation in groundwater composition.

### 3.2. EWQI Modeling

This study computed the suitability of physicochemical quality with the help of the entropy-weighted water quality index (EWWQI) model [25]. They ranged from 39.8 to 138.3 with average of 85.4 shown in Table 4. The descriptive table shows categories of water with its rank that helps to identify the suitability for drinking or domestic purposes. This whole study area belongings to three categories, viz., good (25-50), medium (50-100), and poor (100-150). It has been observed that only one sample found to be in good category of water for drinking. The medium type of category is unfit for drinking purposes while it can be fit for domestic purposes; on other hand, the poor category is neither good for drinking nor for domestic purposes. As illustrated in Figure 2, the 72% of the samples was found in medium category, ranked as 3, 22% of the samples was under poor category, ranked as 4, and only 6% of sample was fall in good category, ranked as 2. The spatial map of EWQI value shown in Figure 3, this picture, clearly shows that the good (EWQI < 50) and medium (EWQI ranged 50-100) quality of water was identified in the center of the research area while the poor (EWQI > 100) quality of water in the eastern part.  Figure 4 shows the percentage of groundwater samples in different category.

### 3.3. Spatial Distribution Map of Heavy Metal

The concentration levels of heavy metals in the region differ significantly. The higher concentration range of manganese (0.0057- 0.14 ppm) was reported in the study area, followed by iron concentration range of (0.0036-00.53 ppm) and arsenic (0.042-0.108), which exceeded the permissible limit prescribed given by the Word Health Organization [23]. Figures 5(a)–5(f) represent spatial distribution map of GIS-based inverse distance weightage (IDW) technique for the pattern of arsenic (As), copper (Cu), manganese (Mn), nickel (Ni), lead (Pb), and iron (Fe). Except in the southeastern and northern zone, the amount of arsenic was found to be dominant across the field of study. The greater level of arsenic in this region could be owing to industrial wastewater discharge into the open ground, contaminating groundwater through infiltration [27]. Furthermore, as a result of chemical weathering, archaean consolidated granite-gneiss rocks of Chotanagpur, which are made up of quartzite and schist, might be the sources of As in this area's groundwater aquifers. Only the research area's southeastern corner is within the arsenic safe contamination zone (Figure 5(a)). Iron (Fe) and manganese (Mn) are naturally available in the earth's crust, and if they exceed the recommended limit, they can cause a variety of issues in groundwater [28]. The map shows the concentration of Fe more in the center and southern parts of the studied region (Figure 5(b)). The Fe contour map in this place can be linked to the earth's crust and the research area's geological development [29]. Mn is an essential element that plays a role in a number of important component [30]. The higher value of Mn was found in some locations of the northern and southern region of study area (Figure 5(c)). The map of Ni, Pb, and Cu demonstrated that throughout the area of research, all three elements are typically within the safe drinking zone (Figures 5(d)–5(f)).

### 3.4. Assessment of Human Health Risks

Oral intake was utilized to determine the health risk of heavy metals in groundwater at all 18 locations. Furthermore, the HI value ranges from 10 to 25 for the study area. Its value is greater than unity because of the major contribution of As, which indicates a very high chronic risk. In contrast, the carcinogenic risk associated with As was found to be <0.1, which indicates less carcinogenic risk. According to the spatial map of HI, the majority of the study region are at a noncarcinogenic risk that might cause significant health problems (Figure 6). The only section of the study area where health risks are minimal is the southeast. It has also been revealed that students are more vulnerable than adults to the danger of heavy metals when consumed orally (Table 5).

The average arsenic concentration was found to be 42.8 ppb to 108 ppb, the carcinogenic risk value shown in Table 6. The concentration of arsenic was found higher in the northern part of the study area which might be due to anthropogenic sources like mining, use of pesticides, and industries located nearby. The excess of arsenic present in groundwater causes arsenicosis diseases as shown in Figure 7 which is now a days very serious issues. Also, it was found that children are at more prone than adult as cancer risk value was higher.

### 3.5. PCA Analysis

The link between the parameters and the principal components was determined using principal component analysis (PCA). The primary components were restricted when the eigenvalue was more significant than 1.  Figure 8 shows a scree plot of the PCA. As a result of the investigation, two major components were identified. These two variables accounted for a maximum of the variance in the data. Arsenic explains the most variation among the metal characteristics, accounting for 37%, while nickel and manganese account for 23% and 20.8 percent of the overall variation. Cu and Fe showed the strongest positive ties to PC1, while Ni had the strongest negative ties to PC1. Cu and Fe exhibited the strongest positive relationship in PC1 and PC2, while Mn and Zn had the most negative relationship. In PC1 and PC2, the relationship between the parameters revealed that Cu > Fe > As > Mn > Zn > Ni and Fe > Cu > Ni > As > Zn > Mn evolved from very positive to strongly negative. Furthermore, a scree plot graph was produced between eigenvalue and principal component number and demonstrated that As (2.24) had the highest eigenvalue while cu had the lowest (0.19). Similar trends of the percentage of variance are shown as eigenvalue.  Table 7 depicts the PCA analysis of metal parameters.

### 3.6. HCA Analysis

Based on metal values, hierarchical cluster analysis was utilized to analyze the closeness and homogeneity inside the sampling sites. The mean correlation resulted in the dendrogram displayed in Figure 9. There are four types of clusters majorly divided shown in different colors, viz., red (Nos. 1,2,6,15, and 16), green (Nos. 910,11,14, and 17), blue [6, 14, 18, 31], and cyan (Nos. 4,7, and 18). Furthermore, the red and green sampling locations formed a subcluster linked with the subcluster of green and cyan to complete the dendrogram linkage. It was also discovered that there was a high correlation between 6, 10, and 12 sampling stations. The 6, 11, and 7 sampling stations revealed significant diversity in which each station exhibited a shaky connection on its own.

### 3.7. Strategy Requires for Groundwater Management

The management of groundwater deals with the complex interaction between the physical environment and human activities. It possesses an extremely difficult challenge for solving the benefit of all parties involved. The rapid urbanization and growing population results in the exploitation of underground water pockets. Consequently, there are rivalries between the exploiters without care about management programs. The management strategies for groundwater management are as follows:

- Groundwater management awareness for beneficiaries
- Limit the exposition according with monitoring results
- Enhancement in the ground water recharge from other sources
- Maintain and avoidance of the degradation of groundwater quality
- Maintaining the minimum level of groundwater especially in unconfined aquifers

## 4. Conclusion

EWQI modeling and hydrogeochemical evaluation could help to evaluate factors controlling chemistry and suitability of groundwater for drinking purposes in Ranchi city. Only 6% of the sample is good quality, while the rest ranges from medium (72%) to poor (3.22%). The concentration level of Mn (0.0057-0.14 ppm), Fe (0.0036-00.53 ppm), and As (0.042-0.108 ppm) exceeds the prescribed guideline by WHO. Through oral intake, children are more susceptible to the risk than adults. Hydrogeochemical processes of groundwater were dominated by reverse ion exchange. The arsenic was the most influencing parameter among all other metals, as its value of HQ > 1.The cluster analysis identified four clusters based on groundwater quality data sets. The study is helpful to avoid the possibility of increasing contamination of groundwater and in ensuring public safety. Since numerous factories are located in this region, carcinogenic risk assessment the other heavy metal that leading to carcinogenic risk must be examined to understand the better influencing heavy metals.

## Figures and Tables

**Figure 1:** Sampling location of the study area.

**Figure 2:** Schematic layout of methodology involved in present study.

**Figure 3:** Spatial distribution of the EWQI model.

**Figure 4:** Percentage of groundwater samples in different categories.

**Figure 5:** (a)–(f) Spatial distribution map of concentration of heavy metal: (a) As, (b) Mn, (c) Fe, (d) Cu, (e) Ni, and (f) Zn.

**Figure 6:** Spatial distribution map of hazard index (HI).

**Figure 7:** Effect of arsenic in human body parts.

**Figure 8:** Scree plot of PCA.

**Figure 9:** Dendrograph of HCA.

**Table 1:** Classification standards of groundwater quality according to Entropy Weighted Water Quality Index (EWQI).

Sl no.	Range of EWQI	Category
01	<25	Excellent
02	25-50	Good
03	50-100	Medium
04	100-150	Poor
05	>150	Unfit

**Table 2:** Carcinogenic risk level scale [26].

Risk level	HQ/HI	Occurrence of cancer	Carcinogenic risk
1	<0.1	<1 per 10 lakh inhabitants	Very low
2	≥0.1 < 1	> 1 per 10 lakh inhabitants <1 per 1 lakh inhabitants	Low
3	≥1 < 4	> 1 per 1 lakh inhabitants <1 per 10 thousand inhabitants	Medium
4	≥ 4	> 1 per 10 thousand inhabitants <1 per inhabitants	High

**Table 3:** The analyzed data of groundwater quality variables.

Parameters	Min	Max	Avg	SD	BIS [24]
pH	7	8.1	7.55	0.31	6.5–8.5
EC	236	1369	554.72	333.57	—
TDS	236	1168	573.05	273.59	500-2000
F^−^	0.21	0.96	0.55	0.25	1-1.5
Cl^−^	31.12	228.3	91.46	59.32	250-1000
HCO_3-_	89	536	222.93	107.31	200-600
SO_4_^−2^	12.6	85.3	42.33	21.83	200-400
NO_3-_	4.1	65.7	24.95	18.10	45
Ca^2+^	22.6	130.6	70.66	30.63	75-200
Mg^2+^	11.8	60.5	33.40	14.35	30-100
Na^+^	12.5	42.3	25.68	9.51	200
K^+^	3.6	18.6	8.46	4.33	12
Total hardness	105.66	578.58	307.54	121.71	200–600

All parameters are in mg/l, except EC(*μ*S/cm) and pH has no unit.

**Table 4:** Categorization of EWQI and its suitability.

Sampling no.	EWQI	Category	RANK	Suitability for drinking purposes	Suitability of domestic purpose
1	39.8	G	2	Fit	Yes
2	45.9	M	3	Unfit	Yes
3	64.9	M	3	Unfit	Yes
4	82.7	M	3	Unfit	Yes
5	61.7	M	3	Unfit	Yes
6	85.4	M	3	Unfit	Yes
7	91.1	M	3	Unfit	Yes
8	134.1	P	4	Unfit	NO
9	138.3	P	4	Unfit	NO
10	107.0	P	4	Unfit	NO
1	74.6	M	3	Unfit	Yes
12	90.5	M	3	Unfit	Yes
13	103.7	P	4	Unfit	NO
14	84.7	M	3	Unfit	Yes
15	73.5	M	3	Unfit	Yes
16	84.2	M	3	Unfit	Yes
17	75.4	M	3	Unfit	Yes
18	99.6	M	3	Unfit	Yes

G: good; M: medium; P: poor.

**Table 5:** HQ value of noncarcinogenic risk of heavy metal.

Sl. no.	AS (xE+01)		NI (xE-02)		Mn (xE-02)		Fe (xE-04)		Zn (E03)		Cu (xE-04)		HI (xE+01)	
	A	C	A	C	A	C	A	C	A	C	A	C	A	C
1	0.98	1.08	2.8	3.3	1.64	1.95	3.46	4.11	4.20	4.99	5.03	5.98	0.93	1.08
2	0.93	1.11	10.9	12.9	0.33	0.39	4.02	4.77	4.56	5.41	5.84	6.93	0.94	1.12
3	1.55	1.84	4.8	5.8	5.72	6.79	3.74	4.44	12.76	15.15	5.44	6.45	1.561	1.85
4	1.45	1.72	9.8	11.6	3.54	4.20	3.46	4.11	11.28	13.38	5.03	5.98	1.47	1.74
5	1.59	1.89	6.2	7.4	5.03	5.97	3.46	4.11	12.80	15.19	5.03	5.98	1.60	1.90
6	1.29	1.53	10.9	12.9	0.50	0.59	4.43	5.26	11.83	14.04	6.44	7.65	1.30	1.54
7	0.83	0.98	3.2	3.8	3.04	3.61	4.29	5.10	14.09	16.72	6.24	7.41	0.83	0.99
8	2.10	2.49	20.4	24.2	5.64	6.70	4.29	5.10	6.62	7.86	6.24	7.41	2.12	2.52
9	1.33	1.58	27.6	32.8	0.60	0.71	3.74	4.44	6.17	7.33	5.44	6.45	1.36	1.62
10	1.30	1.55	28.9	34.3	0.24	0.28	3.46	4.11	4.78	5.68	5.03	5.98	1.33	1.58
11	1.12	1.33	25.8	30.6	0.51	0.61	4.15	4.93	11.60	13.77	6.04	7.17	1.14	1.36
12	1.22	1.45	15.6	18.5	4.96	5.89	3.74	4.44	5.49	6.52	5.44	6.45	1.24	1.47
13	1.79	2.12	20.6	24.5	5.74	6.81	4.43	5.26	6.82	8.09	6.44	7.65	1.82	2.16
14	1.11	1.32	22.8	27.0	1.31	1.55	3.88	4.60	5.85	6.94	5.64	6.69	1.14	1.35
15	1.51	1.79	9.6	11.4	1.13	1.34	4.15	4.93	5.27	6.25	6.04	7.17	1.52	1.80
16	1.31	1.56	3.9	4.6	1.09	1.29	3.46	4.11	4.33	5.14	5.03	5.98	1.32	1.56
17	0.913	1.08	25.1	29.8	1.65	1.96	3.05	3.62	5.43	6.44	4.43	5.26	0.94	1.12
18	1.40	1.66	18.1	21.5	3.15	3.74	3.03	3.60	10.57	12.55	6.14	7.29	1.42	1.69

**Table 6:** The carcinogenic risk value of arsenic(As).

Sample no.	Carcinogenic risk value (adult) (E-03)	Carcinogenic risk value (child) (E-03)
1	4.09	4.85
2	4.20	4.99
3	6.97	8.27
4	6.53	7.75
5	7.15	8.49
6	5.79	6.87
7	3.74	4.44
8	9.44	11.20
9	6.01	7.13
10	5.86	6.96
11	5.02	5.96
12	5.50	6.52
13	8.06	9.56
14	5.00	5.94
15	6.79	8.06
16	5.90	7.01
17	4.11	4.88
18	6.29	7.47

**Table 7:** PCA analysis of heavy metal concentration.

Parameter	Coefficients of PC1	Coefficients of PC2	Eigenvalue	Percentage of variance	Cumulative variance
As	0.42454	-0.18525	2.24	37.48	37.4
Ni	-0.1321	0.42347	1.40	23.47	60.9
Mn	0.40861	-0.53642	1.21	20.23	81.1
Fe	0.48102	0.47852	0.66	11.14	92.3
Zn	0.35787	-0.28842	0.27	4.51	96.8
Cu	0.52527	0.4318	0.19	3.18	100.0

## Data Availability

All the data will be made available on request.
